# ZOMEC via the p-Akt/Nrf2 Pathway Restored PTZ-Induced Oxidative Stress-Mediated Memory Dysfunction in Mouse Model

This article has been retracted.

**DOI:** 10.1155/2022/8902262

**Published:** 2022-09-19

**Authors:** Rifat Jahan, Mohammad Yousaf, Hamayun Khan, Nousheen Bibi, Musarrat Ijaz, Touseef Rehan, Shahid Ali Shah

**Affiliations:** ^1^Department of Chemistry Islamia College University, Peshawar 25120, Pakistan; ^2^Department of Biochemistry, Shaheed Benazir Bhutto Women University, Peshawar, Pakistan; ^3^Department of Bioinformatics, Shaheed Benazir Bhutto Women University, Peshawar, Pakistan; ^4^Department of Statistics, Shaheed Benazir Bhutto Women University, Peshawar, Pakistan; ^5^Department of Food and Nutrition, Shaheed Benazir Bhutto Women University, Peshawar, Pakistan; ^6^Neuro Molecular Medicine Research Center Peshawar, Pakistan

## Abstract

A new mechanistic approach to overcome the neurodegenerative disorders caused by oxidative stress in Alzheimer's disease (AD) is highly stressed in this article. Thus, a newly formulated drug (zinc *ortho*-methyl carbonodithioate (ZOMEC)) was investigated for five weeks on seven-week-old BALB/c male mice. ZOMEC 30 mg/kg was postadministered intraperitoneally during the third week of pentylenetetrazole (PTZ) injection. The brain homogenates of the mice were evaluated for their antioxidant potential for ZOMEC. The results including catalase (CAT), glutathione S transferase (GST), and lipid peroxidation (LPO) demonstrated that ZOMEC significantly reverted the oxidative stress stimulated by PTZ in the mouse brain. ZOMEC upregulated p-Akt/Nrf-2 pathways (also supported by molecular docking methods) to revoke PTZ-induced apoptotic protein markers. ZOMEC reversed PTZ-induced neuronal synapse deficits, improved oxidative stress-aided memory impairment, and inhibited the amyloidogenic pathway in mouse brains. The results suggested the potential of ZOMEC as a new, safe, and neurotherapeutic agent to cure neurodegenerative disorders by decreasing AD-like neuropathology in the animal PTZ model.

## 1. Introduction

Alzheimer's disease (AD) in the brain has been accounted to possess a huge amount of oxidative stress and burden accompanied by the accumulation of both amyloid-beta (A*β* as plaques) and hyperphosphorylated protein [1]. As per reported literature, several metals such as zinc, iron, and copper have a key role in amyloid accumulation and neurodegeneration [2]. Smart studies have reported that both copper and zinc can bind firmly with the N-terminal metal-binding domain of A*β* and its precursor proteins [3, 4]. Moreover, a huge amount of zinc is involved both in memory and cognitive sites of the brain especially the hippocampus being severely damaged during observing AD features [5, 6]. At physiological conditions, there is a balance between the reactive oxygen species (ROS) and antioxidants, but it could be damaged by severity of ROS which makes antioxidant defense less efficient; thus, neurodegeneration occurs and results in cell death [7]. These oxidative and antioxidative mechanisms are balanced by certain molecules, such as nuclear factor erythroid 2-related factor-2 (Nrf-2) and heme oxygenase-1 (HO-1) in normal conditions. Briefly, when Nrf-2 is exposed to oxidative stress, it is transported to the nucleus where it initiates antioxidant mechanisms [8]. This translocation of Nrf-2 results in the transcription of several antioxidant proteins like heme oxygenase-1 (HO-1), glutathione (GSH), and catalase to spread the oxidative stress and protect the cell from apoptosis and inflammation [9, 10]. Further, phosphorylated Akt is regarded as a signal of cell growth and antiapoptosis, while its reduced levels increase the apoptosis by enhancing proapoptotic BAX and BAX/Bcl-2 ratios [11]. A proapoptotic BAX protein that damages the mitochondrial outer membrane and releases cytochrome C activates caspases and finally damages PARP-1 production [12–14]. An antiapoptotic Bcl-2 protein is associated with the outer membrane of mitochondria and can reduce the release of cytochrome C [15]. So the elevated oxidative stress induces cellular abnormalities, impairs the DNA, and leads to dysfunction of mitochondrial energy production, all of which may help in the progression of aging processes and neurodegenerative disease [16]. There are several reported agents like organotin complexes, biomaterials, prodrugs, and biocompatible drug carriers to treat and reduce the oxidative stress overcoming the neurodegenerative disorder [17–24].

Several compounds are used as seizure-inducing drugs, i.e., kainic acid, pilocarpine, and pentylenetetrazole (PTZ) [25], where PTZ drug is the most commonly used models for screening antikindling and anticonvulsants. PTZ is a GABA-A antagonist that is noncompetitive [26]. PTZ kindling is reported to cause a change in the level of neurotransmitters (GABA, glutamate, DA, NE, 5-HT, and their metabolites) in the mouse's brains, in addition to decreasing the oxidative stress, neuroinflammation, and neurodegeneration [27, 28]. Nerve cell death is an energy-dependent molecular cascade process that is highly ordered and involves new gene transcription. An increase in oxidative stress is involved in abnormal nerve function. On the other hand, cell apoptosis occurs in AD. Caspases and BCl2 proteins are two major families that lead to nerve cell death in neurodegenerative diseases [29]. Donepezil (Aricept) is a drug that is used for the treatment of all the stages of AD. Galantamine (Razadyne) and rivastigmine (Exelon) are approved for the treatment of AD patients (mild to moderate). Besides these, memantine extended release and donepezil (Namzaric), memantine (Namenda), azeliragon, pioglitazone, troriluzole, zagotenemab, intepirdine, lumateperone, suvorexant, and aripiprazole are used to treat AD patients [30].

Previous reports recommend that AD affects the endogenous defense system of the body by decreasing the antioxidant concentration. When the antioxidant system of an organism fails to overcome oxidative stress, cellular damage occurs and oxidants accumulate principally in the mitochondria [31]. It is well known through various studies that the oxygen radicals are removed from the body and the cells are rescued by antioxidants such as superoxide dismutase (SOD). Researchers have emphasized and found good results after developing safe and effective antioxidants that could help to prevent neurodegenerative diseases. Considering such neurodegenerative diseases, the therapeutic potential of ZOMEC as a neuroprotective and antioxidative agent was evaluated by using PTZ-induced oxidative stress in BALB/c mice.

The current study is aimed at investigating the new therapeutic agent; ZOMEC was evaluated in reducing PTZ-induced ROS-mediated neuronal synapse deficits, memory and cognition, and A*β* in the brain of mice.

## 2. Materials and Methods

### 2.1. Preparation of ZOMEC

ZOMEC was prepared as per the reported procedure mentioned in Figure SI (supplementary materials) [32].

### 2.2. Animals and Drug Treatment

The solutions were prepared in a saline solution of 0.9% while ZOMEC (administered after the third week on daily basis) was dissolved in DMSO and diluted with saline water (0.9% NaCl). Each mouse group was intraperitoneally (I.P.) injected. The control group was injected with normal saline only. The experimental procedures were performed with all the measures established by the Ethics Committee of the NMMRC (Neuro Molecular Medicine Research Center reference no. 22/2020) according to the guidelines of NIH (International Institute of Health, USA). Seven-week-old BALB/c male mice were selected for the experiments. The treatment groups included a control group (saline), PTZ group (35 mg/kg BW), PTZ+ZOMEC group (35 mg/kg BW and 30 mg/kg BW, respectively), and ZOMEC group (30 mg/kg BW). PTZ was administered on alternative days for five weeks intraperitoneally.

### 2.3. Behavioral Tests

#### 2.3.1. Morris Water Maze (MWM)

MWM test was performed to evaluate the long-term memory and spatial learning of the mice [33].

#### 2.3.2. Y-Maze (YM)

The YM test was performed to study the mouse's exploratory behavior [33].

### 2.4. Collection of Brain Tissue

After five weeks of PTZ and ZOMEC treatment, the animals (*n* = 5/group) were sacrificed (chloroform was used to anesthetize mice). The brains were dissected, and the required cortical brain parts were carefully removed and placed in a Petri dish containing phosphate buffer saline (PBS) and RNA wait in a 1 : 1 solution for about sixty seconds and then frozen in dry ice.

### 2.5. Antioxidant Activity of ZOMEC

#### 2.5.1. Glutathione S Transferase (GST) Level

GST activity was measured using 1-chloro-2,4-dinitrobenzene (CDNB). Each well was filled with a mixture of 1 mM CDNB (10 *μ*L), 5 mM reduced glutathione (10 *μ*L), buffer solution (270 *μ*L), and the sample (10 *μ*L). The absorbance was noted at 340 nm [34]. The kit used was GST catalog no. AB3282 (Sigma-Aldrich).

#### 2.5.2. Catalase Activity

Sigma-Aldrich kit (Cat. C0979) was used to determine catalase activity. To 50 mM sodium phosphate buffer (340 *μ*L) at pH 7.0, the brain tissue supernatant (100 *μ*L) was added. The mixture was incubated for five minutes with 2 M H_2_O_2_ (150 *μ*L). Absorbance was noted at 240 nm for three minutes [35].

#### 2.5.3. Determining Concentration of Lipid Peroxidation

In the current study, LPO assay kit catalog no. MAK085 was used. Malondialdehyde level of the mouse brain was found by boiling a mixture of the brain tissue supernatant (100 *μ*L), 8.1% of SDS solution (100 *μ*L), 20% of acetic acid (375 *μ*L), and 0.25% of thiobarbituric acid (1 mL of TBA) for 1 h. After boiling, 200 *μ*L of the mixture was pipetted into a ninety-six-well plate, and absorbance was noted at 532 nm. MDA levels were extrapolated from the MDA standard curve of plotted concentrations [34].

### 2.6. Western Blot Analysis

The brain tissues were homogenized in 0.01 M PBS containing a protease inhibitor cocktail. After centrifugation, the protein samples were subjected to quantification and were run through SDS-PAGE on 15% gels under reducing conditions and then shifted onto a polyvinylidene fluoride membrane (PVDF). The broad range protein marker 10-250 KD (Precision Plus Protein Standards, Kaleidoscope, Bio-Rad) was run to find out the molecular weights of the proteins. 5 *μ*L of the primary antibody was taken in 7 mL of Tris buffer saline tween (TBST) solution. Primary antibodies ionized calcium-binding adaptor molecule 1 (Iba-1; sc-32725), glial fibrillary acidic protein (GFAP; sc-33673), nuclear factor-erythroid factor 2-related factor 2 (Nrf-2; sc-365949), heme oxygenase (HO-1; sc-136960), phosphorylated protein kinase B (p-Akt; sc-514032), BCL2-associated X protein (BAX; sc-7480), B cell lymphoma 2 (Bcl2; sc-7382), caspase-3 (CASP3; sc-7272), poly (ADP-ribose) polymerase 1 (PARP-1; sc-8007), and beta-actin (*β*-actin; sc-47778) of manufacturer Santa Cruz USA were applied on PVDF membrane, respectively, by keeping them overnight on an orbital shaker at 4°C. 4 *μ*L of secondary antibody in 20 mL of TBST solution (Blotting Grade Affinity Purified Goat Anti-Mouse IgG (H+L) Horseradish Peroxidase Conjugate, cat. #170-6516, Bio-Rad Laboratories, USA) was used for the detection of the target proteins. The secondary antibody was applied to the membrane and placed on a shaker for three to four hours at room temperature so that it can attach to the primary antibody. The bands of the western blot were visualized using electrochemiluminescence (ECL), a detection reagent (Amersham Pharmacia Biotech, Uppsala, Sweden) [36, 37].

### 2.7. Ligand and Receptor 3D Structures

3D structure of ZOMEC was generated from ChemDraw (http://www.cambridgesoft.com) followed by the geometry optimization. The structure of the p-Akt was taken from the protein data bank (PDB) (https://www.rcsb.org/). The three-dimensional structure of Nrf2 protein was constructed through the homology modeling approach (http://www.rcsb.org) using the I-TASSER server [38].

### 2.8. Molecular Docking

The molecular docking of ZOMEC with Nrf-2 and p-Akt was done by using PatchDock. PatchDock is an algorithm for molecular docking. The input is two molecules of any type: proteins, DNA, peptides, and drugs. The output is a list of potential complexes sorted by the shape complementarity criteria.

### 2.9. Statistical Analysis

Computer support ImageJ version 1.51 by NIH, USA, and Prism 5 by GraphPad Software were used for quantification of bands and preparation of their histograms. The analysis of the data was completed with the help of analysis of variance (ANOVA) followed by Tukey's test. The density values of the data are presented as the mean ± SEM of five mice per group and are representative of three independent experiments. *p* values less than 0.05 were considered to be statistically significant; ^∗^*p* < 0.05, ^∗∗^*p* < 0.01, and ^∗∗∗^*p* < 0.001 indicate comparison between the PTZ and ZOMEC+PTZ groups; ^#^*p* < 0.05, ^##^*p* < 0.01, and ^###^*p* < 0.001 indicate comparison between the control and PTZ groups; ^@^*p* < 0.05, ^@@^*p* < 0.01, and ^@@@^*p* < 0.001 indicate comparison between the control and ZOMEC groups; and ns indicates no significance among the groups.

## 3. Results

### 3.1. ZOMEC Ameliorated Oxidative Stress Markers Induced by PTZ in the Mouse Brain

Previous studies indicated that both CAT and GST are the major antioxidant agents [39]. For this reason, the brain tissue homogenates of mice were analyzed with different antioxidant assays including CAT, GST, and LPO. The results indicated that PTZ significantly inhibited CAT (9 *μ*mol/min/mg of protein) which was increased to 17 *μ*mol/min/mg of protein by the group attenuated with PTZ+ZOMEC in comparison to the control one (25 *μ*mol/min/mg of protein). GST was significantly reduced in PTZ-attenuated mice (12 *μ*mol/min/mg of protein) as compared to the control (44 *μ*mol/minute/mg of protein), while ZOMEC increased the GST levels in the PTZ+ZOMEC group (27 *μ*mol/min/mg of protein) compared with the PTZ group. As far as LPO is concerned, its activity was increased in the diseased mice (120 *μ*mol/min/mg of protein) as compared to the control one (40 *μ*mol/min/mg of protein). In the PTZ+ZOMEC group, the LPO was 65 *μ*mol/min/mg of protein. The group of healthy mice receiving ZOMEC showed no significant difference in LPO (42 *μ*mol/min/mg of protein) compared to the control group (40 *μ*mol/min/mg of protein). However, a statistical difference was seen in CAT (19 *μ*mol/min/mg of protein) and GST (34 *μ*mol/min/mg of protein) as compared with the control group (25 *μ*mol/min/mg of protein and 44 *μ*mol/min/mg of protein, respectively) (Figures 1(a)–1(c)).

### 3.2. ZOMEC Inhibited PTZ-Activated Glial Cell Activation in the Mouse Brain

PTZ can activate the glial cells in adult male mouse brains [40]. The current study similarly found that the male mice that were attenuated with PTZ significantly increased the protein expression of microglia (Iba) and astrocytes (GFAP) compared with the control group, while the PTZ+ZOMEC inhibited the expression of both the proteins to a significant level compared with the PTZ group as shown in Figures 2(a)–2(c). The ZOMEC group when compared to the control group showed no significance in the protein expression of Iba-1 and GFAP.

### 3.3. ZOMEC Attenuated Mouse-Reversed PTZ-Induced Neuroapoptosis/Neurodegeneration

The previous reports confirmed that neuronal cell death due to PTZ is apoptotic death [31]. To confirm this statement, the brain homogenates of the selected groups were used through western blot analysis. The results showed that PTZ activated the apoptotic cascade and enhanced the expression of caspase-3, BAX, and PARP-1 proteins. It considerably downregulated Bcl2 protein and increased BAX/Bcl2 ratio in the homogenates of mouse brains compared with the control group. Interestingly, the test compound ZOMEC treatment in the PTZ+ZOMEC group not only reduced the proteins caspase-3, BAX, and PARP-1 but also decreased BAX/Bcl2 ratio compared with the PTZ group. The ZOMEC group significantly reduced BAX and Bcl2 and increased PARP-1 compared with the control group. However, no significant difference was noticed in BAX/Bcl2 and caspase-3 when compared with the control group as depicted in Figures 3(a)–3(f).

### 3.4. ZOMEC Abrogated PTZ-Induced Amyloidogenic A*β* Pathways in Mice

A*β* and BASE1 have been shown to increase in neurodegenerative diseases [28]. The level of BACE1 and A*β* proteins was investigated through western blot analysis. The results indicated that PTZ induction significantly upregulated the A*β* and BACE1 protein activity in the mouse brain compared with the control group. The PTZ+ZOMEC-induced mouse group significantly lowered the BACE1 and A*β* (amyloidogenic pathway) expression compared with the PTZ group. In the ZOMEC group, no significant difference was seen in BACE1 and A*β* compared with the control mice as shown in Figures 4(a)–4(c).

### 3.5. ZOMEC Treatment Improved Pre- and Postsynapse Protein Production in PTZ-Induced Mice

The synaptic abnormalities that arise in the hippocampus are associated with cognitive impairment. Presynaptic, i.e., synaptophysin (SYP), and postsynaptic, i.e., postsynaptic density protein (PSD-95), proteins play an important role in these synaptic abnormalities [41]. In the current study, the comparative expression of SYP and PSD-95 in the brain homogenate of the selected mouse groups was analyzed through the western blot. The expression of both the proteins significantly increased in the brain of PTZ+ZOMEC group mice, while PTZ-induced mice were noted with a decreased protein concentration of SYP and PSD95 as shown in Figures 5(a)–5(c).

### 3.6. ZOMEC Rectified PTZ-Induced Memory Dysfunction in Mice

The effect of ZOMEC on long-term memory and spatial learning in AD (PTZ-induced) mice was estimated through MWM. To find the submerged target, the mean latency decreased gradually in selected groups. On the first day of the behavior test, the immersed target was found in sixty seconds by the PTZ-administered mouse group while the mice with the compound ZOMEC (30 mg/kg) along with PTZ (35 mg/kg) found it in twenty-eight seconds. ZOMEC-treated mice found the platform in thirty-nine seconds and the control group in twenty-three seconds. On the subsequent days, the PTZ-attenuated group finished the task of the immersed target. But the mean escape latency (seconds) was found greater for the PTZ-administered group compared to the other experimental mouse groups as shown in Figure 6(a).

Further probe test was performed (when the target stand was absent), and the data was recorded on day six. Data collected showed that the PTZ group mice spent time more in the respective quadrant in comparison to the control group. ZOMEC+PTZ group mice spent twelve seconds during the probe test, while no significance was seen in the ZOMEC group compared with the control group (Figure 6(b)). The Y-maze resulted in a significant increase in percent spontaneous alteration in the PTZ+ZOMEC AD mice compared with the control group. On the other hand, the PTZ group resulted in reduced percent spontaneous alteration, while no significance was observed in the ZOMEC group when compared with the control group (Figure 6(c)).

### 3.7. ZOMEC Stimulated p-Akt/Nrf-2 Signaling Pathways

Nrf-2 and HO-1 are said to be the protection systems in the body that are antioxidative. Their level decreases due to an increase in oxidative stress [42]. Being an antioxidant, the protein (Nrf2 and HO-1) expression was checked through western blot analysis. Results indicated that PTZ decreased both the proteins to a greater extent in PTZ-induced AD mice compared to the control group. The PTZ+ZOMEC group showed an increase in protein expression significantly as compared with PTZ, while the ZOMEC group showed no significance in the case of Nrf-2 and increased the level of HO-1 as compared with the control group. Further, western blot analysis resulted in a decreased level of p-Akt in AD mouse brains compared to control, while the PTZ+ZOMEC group showed an increase in p-AKT expression compared with the PTZ group. A significant rise was seen in the ZOMEC group compared with the control as shown in Figures 7(a)–7(d).

### 3.8. Bioinformatics Analysis

To find the role of the compound ZOMEC in AD mice, its binding was visualized with p-Akt through molecular docking. Through docking analysis, the binding of ZOMEC with the p-Akt active site was found with a binding free energy of -13.30 (Table 1). VAL270, TYR272, and ASP292 made conventional hydrogen bonds with ZOMEC apart from several hydrophobic interactions by ASN54 and THR82 amino acids (Figure 7(e), Table 1). The computational analysis further supported the wet laboratory western blot experiments, in which ZOMEC stimulated the p-Akt protein. The experimental results found through western blot recommended that ZOMEC stimulated the Nrf2 signaling pathway (present in the cytoplasm with keap1). The molecular docking analysis of ZOMEC and Nrf2 was carried out to evaluate whether ZOMEC binds to Nrf2 and makes possible its movement towards the nucleus. Docking analysis revealed that ZOMEC binds with the Nrf2 active site with the binding free energy of -8.59 (Table 1). GLU427, GLN411, and LEU407 make conventional hydrogen bonds with ZOMEC apart from several hydrophobic interactions with VAL319, GLY412, THR415, and PRO426 amino acids (Figure 7(f), Table 1).

The table shows global energy, attractive VdW, hydrogen bonding, and hydrophobic interaction of ZOMEC with p-Akt and Nrf2. The results showed that p-Akt and Nrf2 have strong interaction with ZOMEC, which increases their efficacy and helps in curing PTZ-induced neurodegeneration. The computational analysis supported our western blot experiments in which ZOMEC stimulated the Nrf2 protein. Nrf2 translocates into the nucleus to bind to antioxidant-responsive elements in genes encoding antioxidant enzyme heme oxygenase-1 (HO-1). The increased expression of this enzyme plays a key role in mediating cellular detoxification, antioxidation, and anti-inflammatory effects.

## 4. Discussion

The therapeutic potential of ZOMEC as a neuroprotective and antioxidative agent was evaluated by using PTZ-induced oxidative stress in BALB/c mice. It has been proven through the results that ZOMEC treatment upregulated CAT and GST and downregulated LPO as shown in Figures 1(a)–1(c). Thus, ZOMEC considerably decreased oxidative stress in adult mouse brains, consistent with the previous study [43]. Some heavy metals, such as cadmium and nickel, have been reported with toxic levels causing damage to the brain and other organs of the body [22, 24]. When these metals exceed a certain level within the body, their first targeted organelle is mitochondria. Their toxic effect includes oxidative damage to the cells, stunted growth, overexpression of genes, abnormal biochemical and physiological changes, altered behavior, and inadequate metabolism [17].

The study confirms that ZOMEC treatment of mice results in increased SYP and PSD95 protein expressions. In consecutive five days of behavior test, the mean escape latencies of the adult mice were lowered in finding the immersed target. The mice in the control group exhibited a decrease in mean escape latency. It can be figured out in Figure 6(a) that the mouse group treated with PTZ resulted in longer escape latencies compared with the control group. The results specified that spatial learning dysfunction and memory impairment take place in PTZ-attenuated male albino mice. The PTZ+ZOMEC group appreciably decreased the escape latencies to the target compared with the PTZ-administered mouse group. The current study revealed that ZOMEC significantly increased Nrf-2/Ho-1 protein expression in mouse groups. These results were also supported by the docking results shown in Figure 7.

The proposed schematic diagram shows the mechanism of action of ZOMEC as shown in Figure 8. The test compound ZOMEC showed an increased survival pathway of the cell by increasing the expression of p-Akt/Nrf2 proteins. A large increase in Iba-1 GFAP, p-Akt, Nrf2, and BAX/Bcl-2 proteins was noted.

The diagram shows how PTZ induces its toxic effect by inhibiting p-Akt/Nrf-2 signaling pathways. The effect of ZOMEC on the expression of proteins is shown with a green arrow while the protein results found after PTZ administration are shown with a red arrow.

## 5. Conclusion

ZOMEC as a therapeutic agent was applied in an animal model to treat neurodisorder caused by oxidative stress. The results verified a decrease in A*β* production, neuroinflammation, and oxidative stress by applying ZOMEC. The expression of protein markers BAX/Bcl2, caspase-3, and PARP-1 was found through western blot. Interestingly, ZOMEC reversed PTZ-induced neuronal synapse deficits, improved oxidative stress-aided memory impairment, and inhibited the amyloidogenic pathway in mouse brains. Thus, ZOMEC might be one of the first-choice drug candidates to treat AD and associated diseases next-generation neurotherapeutics.

## Figures and Tables

**Figure 1:** ZOMEC reduced PTZ-induced oxidative stress. Shown are the different antioxidant enzyme assays including (a) CAT, (b) GST, and (c) LPO. Significance: ^###^*p* ≤ 0.001, ^∗∗^*p* ≤ 0.01, ^@^*p* ≤ 0.05, and ns = no significance.

**Figure 2:** Activated glial cells (PTZ-induced) were deactivation by our test drug ZOMEC. (a) Shown are the immunoblots of glial cells, Iba-1 and GFAP (both microglia and astrocytes). (b) Histogram of microglia. (c) Histogram of astrocytes. Significance: ^##^*p* ≤ 0.01, ^∗∗^*p* ≤ 0.01, and ns = no significance.

**Figure 3:** ZOMEC reduced PTZ-induced neuroapoptosis in adult mice. Shown are the different apoptotic protein markers including (a) immunoblot of BAX, Bcl2, BAX/Bcl2, caspase-3, and PARP-1, while histograms of all the markers are shown as (b) BAX, (c) Bcl2, (d) BAX/Bcl2, (e) caspase-3, and (f) PARP-1. Significance: ^###^*p* ≤ 0.001, ^##^*p* ≤ 0.01, ^∗∗∗^*p* ≤ 0.001, ^∗∗^*p* ≤ 0.01, ^@^*p* ≤ 0.05, ^@@@^*p* ≤ 0.001, and ns = no significance.

**Figure 4:** ZOMEC significantly downregulated A*β* accumulation and BASE1 production in mouse brains. Shown are the western blot results of A*β* and BACE1. (a) Immunoblot of A*β* and BACE1. (b) Histogram of A*β*. (c) BACE1. These representative bar graphs show the relative density of proteins in the selected groups. Significance: ^###^*p* ≤ 0.001, ^∗∗^*p* ≤ 0.01, and ns = no significance.

**Figure 5:** ZOMEC increased SYP and PSD95 activities in the brain (*n* = 5 animals/group). (a) Immunoblot of SYP and PSD95. (b) The histogram shows a significant increase of SYP levels in the PTZ+ZOMEC group. (c) Significant increase of PSD95 activity with the administration of ZOMEC. Significance: ^##^*p* ≤ 0.01 and ^∗∗^*p* ≤ 0.01.

**Figure 6:** ZOMEC successfully reversed PTZ-induced memory dysfunction in mice (*n* = 5 animals/group). (a) Given are the results for mean escape latency of the MWM for all four experimental groups for five days. (b) Probe test: performed during MWM on day sixth when the submerged stand was absent. (c) The percent spontaneous alteration of selected mouse groups in Y-maze. Significance: ^##^*p* ≤ 0.01, ^∗∗∗^*p* ≤ 0.001, ^∗∗^*p* ≤ 0.01, ^@^*p* ≤ 0.05, and ns = no significance.

**Figure 7:** ZOMEC activated the p-Akt/Nrf-2 signaling pathway to decrease neurodegeneration and memory impairment. (a) Immunoblot results for p-Akt and Nrf-2 protein markers. (b) p-Akt histogram. (c) Nrf-2 histogram. (d) HO-1 histogram. (e) Binding mode and interaction of ZOMEC with p-Akt. (e) A: hydrophobic representation of p-Akt protein with bound ZOMEC shown in zoom view. B: p-Akt protein in ribbon representation with binding residues shown in yellow sticks and ZOMEC in red sticks. (f) Binding mode and interaction of ZOMEC with Nrf2. (f) A: hydrophobic representation of Nrf2 protein with bound ZOMEC shown in zoom view. B: Nrf2 protein in ribbon representation with binding residues shown in blue sticks and ZOMEC in red sticks. Significance: ^###^*p* ≤ 0.001, ^∗∗∗^*p* ≤ 0.001, ^∗∗^*p* ≤ 0.01, ^@^*p* ≤ 0.05, ^@@^*p* ≤ 0.01, and ns = no significance.

**Figure 8:** The schematic representation of the proposed pathway followed by ZOMEC.

**Table 1:** ZOMEC (30 mg/kg) activated the p-Akt/Nrf2 pathway by decreasing memory dysfunction.

Receptors	Global energy	Attractive VdW	Hydrogen bonding	Hydrophobic interaction
p-Akt	-33.50	-13.30	^a^VAL270, ^b^TYR272, and ^c^ASP292	^d^ASN54 and ^e^THR82
Nrf2	-26.42	-8.59	^f^GLU427, ^g^GLN411, and ^h^LEU407	^a^VAL319, ^i^GLY412, ^e^THR415, and ^j^PRO426

^a^Valine, ^b^tyrosine, ^c^aspartic acid, ^d^asparagine, ^e^threonine, ^f^glutamate, ^g^glutamine, ^h^leucine, ^i^glycine, and ^j^proline.

## Data Availability

Data will be provided on request.

## Supplementary Materials

Supplementary Materials Preparation of ZOMEC. Solution of zinc chloride dehydrate (1 mmol) in 10 mL methanol was added to a solution of potassium O-alkyl carbonodithioate (1 mmol) in methanol (30 mL) in a two-necked round bottom flask (100 mL) with continuous stirring at room temperature for 4 h. The solvent was evaporated slowly at room temperature; the solid product obtained was filtered off and dried in air. The product was recrystallized in chloroform : n-hexane mixture (1 : 1).  The synthesized compound was confirmed experimentally by nuclear magnetic spectroscopy ^1^H-NMR spectrum of the test drug.
